RETRACTED

# Computed Tomography- (CT-) Based Virtual Surgery Planning for Spinal Intervertebral Foraminal Assisted Clinical Treatment

**DOI:** 10.1155/2021/5521916

**Published:** 2021-03-06

**Authors:** Hao Li, Song Wang, Jinlong Tang, Jibin Wu, Yong Liu

**Affiliations:** Department of Orthopaedics, Affiliated Hospital of Xuzhou Medical University, Xuzhou, Jiangsu 221000, China

## Abstract

With the development of minimally invasive spine concepts and the introduction of new minimally invasive instruments, minimally invasive spine technology, represented by foraminoscopy, has flourished, and percutaneous foraminoscopy has become one of the most reliable minimally invasive procedures for the treatment of lumbar disc herniation. Percutaneous foraminoscopy is a safe and effective minimally invasive spinal endoscopic surgical technique. It fully protects the paravertebral muscles and soft tissues as well as the posterior column structure of the spine, provides precise treatment of the target nucleus pulposus tissue, with the advantages of less surgical trauma, fewer postoperative complications, and rapid postoperative recovery, and is widely promoted and used in clinical practice. In this paper, we can view the location, morphology, structure, alignment, and adjacency relationships by performing coronary, CT, and diagonal reconstruction along the attachment of the yellow ligaments and performing 3D reconstruction or processing techniques after performing CT scans. This allows clinicians to observe the laminoplasty and the stenosis of the vertebral canal in a more intuitive and overall manner. It has clinical significance for the display of the sublaminar spine as well as the physician's judgment of the disease and the choice of surgery.

## 1. Introduction

Lumbar disc herniation (LDH) is a common degenerative disease, mainly manifesting as back and leg pain and sensory abnormalities related to the lower extremities, and its onset has gradually become younger in recent years, affecting the normal life of patients [1–3]. With the continuous progress of medical technology, spinal foraminoplasty has been used in clinical practice, and spinal foraminoplasty has the advantages of less bleeding, less trauma, and faster recovery, with significant clinical effects [4]. In clinical practice, lumbar disc herniation is an orthopedic disease with a high incidence, and the main symptom is back and leg pain, which is mainly caused by degenerative changes in various parts of the lumbar disc, which not only affects the physical and mental health of patients but also seriously affects their quality of life. In recent years, with the change of living environment and the increase of people's life and work pressure, this disease is gradually developing in the direction of youth, so it is necessary to pay attention to lumbar disc herniation and take effective ways to treat it [5]. Surgery is an effective treatment for lumbar disc herniation, but although small incision surgery can achieve good results and a high success rate, patients need to suffer a lot of pain during the surgery and are prone to postoperative complications, such as incision infection, spinal instability, and nerve root compression, and patients usually need a long time to recover and are prone to recurrence [6–8]. Along with the continuous progress and development of medical technology, intervertebral foraminoscopy has been improved and gradually developed as one of the effective and advanced ways to treat patients with lumbar disc prolapse. Spinal intervertebral foraminoscopy uses percutaneous puncture to place the endoscope into the intervertebral foramen, and with the aid of the endoscope, the nucleus pulposus can be removed and there is a repair of the fibrous ring.

RETRACTED

When studying the structure of the human vertebral body, we found that some of the anterior lower lateral margins of the vertebral plate are located in the migration between the inferior pedicle notch and the inferior articular eminence with the tip facing downward, which we refer to as the “sublaminar spine.” The sublaminar spine is located behind the internal opening at the beginning of the intervertebral canal and forms the posterior lateral wall of the spinal canal. The posterior wall of the intervertebral canal is generally considered to consist of the lateral part of the inferior articular process, the lateral part of the ligamentum flavum, the anterolateral aspect of the superior articular process, and the interarticular process [9]. The upper and lower boundaries of the intervertebral foramen are the inferior and superior incisors of the adjacent vertebral body's vertebral roots, the anterior boundary is the intervertebral disc and vertebral body, and the posterior boundary is the articular eminence joint; the intervertebral foramen in the cervical region is in a horizontal position, and the spinal nerve roots in the lumbar region have to travel obliquely downward in the lateral crypt and then exit the intervertebral foramen immediately above the intervertebral foramen. Clinically, the pathway of the spinal nerve roots, including the intervertebral foramen, is called the intervertebral canal. The direction of travel of the nerve roots out of the spinal canal and into the intervertebral canal shows that the nerve roots are immediately anterior to the sublaminar spine and then enter the intervertebral canal, which is the narrowest at the beginning of the intervertebral canal, and the sublaminar spine is part of the beginning of the posterior wall of the nerve root canal, so the shape, size, and direction of the sublaminar spine are important to whether the spinal nerve is compressed. The study of the sublaminar spine has clinical significance because it can narrow the entrance to the intervertebral canal and is involved in the bony lateral posterior wall that makes up the canal and the bony posterior wall of the internal opening of the intervertebral canal, which may compress the spinal cord or nerve roots [10]. Since the composition of the internal orifice of the intervertebral canal and the posterior wall of the spinal canal overlap with the distribution of the sublaminar spine, the sublaminar spine also participates in constituting the internal orifice of the intervertebral canal and the posterior wall of the spinal canal, being part of them, and therefore tends to cause slenderness and narrowing of the intervertebral canal or spinal canal in the corresponding area, causing compression of the nerve roots or spinal cord traveling within it. The shape, alignment, and distribution of the sublaminar spine are different, and the correspondingly caused signs and clinical symptoms are also different, as shown in Figure 1. The distribution and adjacent structures of the sublaminar spine in the thoracic and upper lumbar spine are different from those of the sublaminar spine in the lower lumbar segment. The thoracic and upper lumbar sublaminar spines mainly compress the spinal canal and may produce corresponding symptoms such as lumbago, back pain, lumbar and knee tenderness, weakness and numbness, and stiffness of the extremities, which are similar to the corresponding symptoms and signs of spinal stenosis and nerve compression caused by degenerative changes of the ligamentum flavum and are not easily distinguished clinically. In the lower lumbar segment, the sublaminar spine mainly compresses the intervertebral canal, which usually produces symptoms similar to those of lumbar disc herniation, such as lumbar pain, numbness in the upper and lower extremities, and even claudication. Sometimes, spinal CT examination may reveal that the lumbar disc is not herniated or the herniation is not serious, which may cause some difficulties for clinicians in diagnosis [11]. Therefore, the observation of the sublaminar spine should be taken seriously to provide clinicians with certain side references, and the observation of the alignment, morphology, and position of the sublaminar spine, whether the intervertebral canal is narrowed, and whether there is nerve compression when the patient undergoes lumbar disc CT scan is of certain guiding significance for the clinician's judgment [12–15].

RETRACTED

In this study, patients with lumbar disc herniation were treated with spinal foraminoscopy and compared with small incision surgery. The results showed that the operative time, incision length, bed rest, and hospital stay were shorter in the study group than in the control group, and intraoperative bleeding was less than in the control group. The pain scores on postoperative days 1, 2, 3, and 4 were lower than those of the control group. This shows that spinal foraminoscopy can shorten the operative time, reduce intraoperative bleeding, shorten bed rest and hospital stay, cause no serious trauma to the patient, reduce the patient's pain level, and is beneficial to the patient's postoperative recovery. Therefore, spinal foraminoscopic surgery can be an effective way to treat patients with lumbar disc herniation. In conclusion, the application of spinal foraminoscopy in the treatment of patients with lumbar disc herniation has a definite effect on the postoperative recovery of patients, and it can also lead to pain reduction, which is of significant clinical value. However, there is a lack of observation of long-term efficacy data in patients with lumbar disc herniation treated with spinal foraminoscopy, and there is a certain probability of recurrence, so a regular postoperative review should be performed to prevent recurrence of the disease by avoiding excessive physical labor and being sedentary.

## 2. Related Work

A typical vertebra consists of a vertebral body, a vertebral arch that extends over several projections, and a vertebral foramen that contains the spinal cord, spinal membrane, and blood vessels. Adjacent vertebrae are connected on opposite sides by intervertebral discs. The entire spine and intervertebral discs form the body's strong and bendable central skeleton and support the full weight of the head and torso, even as they transmit the stresses generated by the muscles directly or indirectly associated with them. The vertebral foramina are connected to form the spinal canal, and the vertebral arch is connected to the vertebral body to form the intervertebral foramen, through which pass the spinal nerves, spinal vertebral branches, blood vessels, and lymphatic vessels. The vertebral body is cylindrical in shape, and the vertebral body of the spine varies in size, shape, proportion, and function because of its location. The vertebral arch root is located in the upper posterior lateral part of the vertebral body and is a short, thick, rounded protrusion [16]. There are depressions at the superior and inferior edges of the vertebral arch root, called the superior and inferior vertebral notch, respectively. The margins of the intervertebral foramen consist of the superior and inferior vertebral notches, the posterior lateral portion of the adjacent vertebral body and the dorsolateral aspect of the intervertebral disc, and the joint capsule of the articular eminence joint. The vertebral roots continue posteriorly directly into the vertebral arch, which is flat in the vertical direction and curves medially posteriorly. Pairs of upper and lower synapses emanate from the vertebral plate at the junction of the plate and the pedicle [17–19].

RETRACTED

The superior articular process extends superiorly, and the dorsal articular surface on the superior articular process may be tilted laterally or medially at different segments. The inferior articular process extends inferiorly, and its ventral side forms the articular surface, which also tilts laterally or medially at different segments. The articular eminences of adjacent vertebrae form the articular eminence joint and become part of the posterior border of the intervertebral foramen. The articular eminence allows the limited motion of the spine, and its mobility varies significantly with the spinal segment [20]. The spine lamina vertebrae inferior (SLVI) is a bony prominence located at the junction of the anterior inferior lateral border of the vertebral plate and the upper part of the root of the inferior articular eminence. One view is that the sublaminar spine is a bony prominence formed by degenerative lesions of the outer edge of the intervertebral ligament [21].

The main basis of the above view is that the outermost position of the sublaminar spine is consistent with the lateral edge of the intervertebral ligament, and the ossification of the intervertebral ligament mainly occurs at the small joints where activities are more frequent, such as the vertebral body at the thoracolumbar segment, and the sublaminar spine also occurs there, which coincides with the distribution pattern of the incidence of the sublaminar spine, and the main pathological changes of the degenerative lesions of the ligament are hypertrophy of the ligament, calcification of the ligament, and ossification of the ligament. The literature shows that the elastic fibers of the ligamentum flavum will break and degenerate due to external stress or aging and then repair themselves to limit fibrosis, and over time, the ligamentum flavum will calcify and ossify, so calcification and ossification of the ligamentum flavum are positively correlated with age, small joint degeneration, and stress. The sublaminar spine is closely related to the location of the ligamentum flavum, and the sites with a higher incidence are also those with higher mobility, higher age, and spinal instability; therefore, it is believed that the formation of the sublaminar spine is a bony protrusion formed by further ossification of the intervertebral ligamentum flavum on the basis of strain, degeneration, repeated repair, and hyperplasia [22–24].

RETRACTED

Another view is that the sublaminar spine is a bony structure that occurs normally in the adult spine and is the attachment point of the intervertebral ligament on the vertebral plate. The main basis of this view is that the subvertebral spine is more fixed and connected to the intervertebral ligament, so it is considered to be a normal bony structure as an attachment point of the intervertebral ligament on the vertebral plate. However, the formation of bone tissue requires mesenchymal cells, ossification centers, osteoblasts, etc. The author reviewed the relevant literature and did not find substances such as ossification centers associated with the sublaminar spine in the process of vertebral plate formation; therefore, the author does not consider the sublaminar spine to be a bony structure of the spine. Since the composition of the internal opening of the intervertebral canal and the posterior wall of the spinal canal overlap with the distribution of the sublaminar spine, the sublaminar spine also participates in forming the internal opening of the intervertebral canal and the posterior wall of the spinal canal and is part of them, thus easily causing the slimness and narrowing of the intervertebral canal or spinal canal in the corresponding area and causing compression of the nerve roots or spinal cord traveling within them. The shape, course, and distribution of the sublaminar spine are different, and the corresponding signs and clinical symptoms are also different. The distribution and adjacent structures of the sublaminar spine in the thoracic and upper lumbar spine are different from the sublaminar spine in the lower lumbar segment. The thoracic and upper lumbar sublaminar spines mainly compress the spinal canal and may produce corresponding symptoms such as lumbago, back pain, lumbar and knee tenderness, weakness and numbness, and stiffness of the extremities, which are similar to the corresponding symptoms and signs of spinal stenosis and nerve compression caused by degenerative changes of the ligamentum flavum and are not easily distinguished clinically.

## 3. Interspinal Relationships in Interspinous Foraminoscopic Virtual Surgery

### 3.1. Relationship between the Lumbar Sublaminar Spine and Lumbar Disc Herniation

Lumbar disc herniation is one of the most common diseases in spinal surgery, which refers to the fracture or rupture of the fibrous ring of the lumbar disc due to trauma or degenerative disease, causing the nucleus pulposus and other tissues with reduced elasticity to protrude, prolapse, or bulge posteriorly or externally under the action of certain external forces, causing the corresponding nerve roots to be compressed, resulting in corresponding clinical symptoms, usually leading to low back pain, numbness of one or both lower limbs, or intermittent. It usually leads to symptoms such as low back and leg pain, numbness, or intermittent claudication in one or both lower limbs, and in severe cases, it can affect the patient's work and life. There are various reasons for the onset of lumbar disc herniation, including endogenous factors such as genetics, developmental abnormalities and degenerative changes, and exogenous factors such as repetitive stress injuries, malnutrition, and trauma. Clinically, surgical treatment is generally adopted for patients with indications for surgery. In the daily surgical approach, epidural anesthesia is first taken, the patient is placed in a prone position, the spinous process of the spine is fully exposed, and the paraspinal tissue on the side with relatively severe symptoms and obvious clinical symptoms is selected as a priority, so that the vertebral space is fully and completely exposed, and then the corresponding part of the soft tissue at the lower edge of the lumbar plate is occluded from above, and then the soft tissues on the upper edge of the adjacent vertebral plate were removed from the lower part, followed by cutting open the ligamentum flavum, opening a small bone window at the corresponding location, freeing the corresponding compressed nerve root tissues in the lumbar region to eliminate the compression, scraping away part of the nucleus pulposus in the corresponding vertebral space, widening the originally narrow lateral saphenous fossa to make it wider and allowing the nerve roots to pass at will, and then repairing the fibrous capsule when the nerve compression condition was lifted. After the nerve compression is removed, the surgery is completed by repairing the fibrous capsule.

RETRACTED

The other surgical procedure is a posterior spinal microendoscopic procedure with the same epidural anesthesia, with the patient also in the prone position and with full exposure of the spinal spinous process, but this time with the help of a large instrument, a small incision is made in the posterior spine under C-arm fluoroscopy. The tip of the needle is fixed to the lower edge of the vertebral plate above the diseased spinal segment, and a dilatation tube is placed there to remove the soft tissue outside the vertebral plate and to expose the vertebral plate space on the side of the lesion. An endoscope is placed in the appropriate area and the intervertebral ligament is pushed through the nerve stripper at the point of attachment at the lower edge of the vertebral plate under direct visualization through the endoscope. The ligamentum flavum is pushed away to fully expose the vertebral plate. At this time, the soft tissue on the surface of the vertebral plate is removed to separate the sublaminar ligamentum flavum, and then the intervertebral ligamentum flavum is removed to fully expose the dura mater and nerve roots, as shown in Figure 2. After removing part of the hypertrophied synovium and the intervertebral ligament, the nerve root compression symptoms were reduced and disappeared, the herniated nucleus pulposus was found, and the nucleus pulposus was removed to complete the operation.

In recent years, with the rapid development of science and technology, especially the continuous progress of minimally invasive technology, posterior spinal microendoscopic surgery has gradually become the first choice of clinicians for the treatment of lumbar disc herniation, which helps to relieve the pain of the majority of patients. Compared with traditional open surgery, posterior spinal microendoscopic surgery has the advantages of relatively less damage to the posterior spinal structures, making the stability of the spine less likely to be damaged and also reducing the inflammatory response of the body. However, posterior microendoscopic spine surgery requires a high level of operator skill and has certain limitations and contraindications for patients, such as older age, significant spinal space narrowing, and severe microarticular hyperplasia. At the same time, in order to achieve the desired results, the operating surgeon should keep in mind the relevant intraoperative precautions and needs to fully grasp the anatomical relationship between the inferior spinous process and the sublaminar ridge, as well as the anatomical position of the corresponding intervertebral foramen and the surrounding relationships. Since the distribution of the sublaminar spines is not fixed, most of them will be found around the internal orifice of the intervertebral canal and will have some involvement in the internal orifice of the intervertebral canal and the bony posterior wall of the spinal canal. If the sublaminar spines are large in size, they will cause stenosis of the intervertebral canal and cause the corresponding symptoms. Therefore, the study of the incidence and anatomical location of the sublaminar spine and its adjoining relationship is of vital importance for the treatment of lumbar intervertebral discs by posterior microendoscopic surgery of the spine, which can provide some help to the clinicians.

RETRACTED

### 3.2. The Relationship between the Inferior Spine of the Vertebral Plate and the Ligamentum Flavum

The ligamentum flavum is an important part of the spine, and 70% to 80% of its tissue composition is composed of elastic fibers, mainly longitudinal elastic fibers arranged in a band and collagen fibers mixed in the elastic fibers, which can increase the elasticity of the ligamentum flavum and allow the body to make some movements more naturally, which is very important for maintaining the ability of the spine to posterior extension, forward flexion, and lateral flexion. The elastic fibers can extend under the action of force, even to 1 to 1.5 times their original length, but when the ligament extends beyond its limit or is always in a state of high progression, there is a possibility of sudden rupture. Collagen fibers can prevent excessive stretching and deformation of elastic fibers and prevent rupture. Elastin fibers are composed of a core of elastin and are covered with microfibers. The action of the microfibers allows the elastin to become fibrous, enabling the intervertebral ligament to withstand the force.

Along with the ossification of the intervertebral ligament, the structure of the ligament undergoes great changes, in which the regularly arranged elastic fibers are replaced by collagen fibers in a haphazard arrangement, and the ligament also contains fibroblasts and chondrocytes, which create the conditions and basis for the degeneration and ossification of the ligament. Physiological and pathological degeneration of the ligamentum flavum, such as calcification, ossification, and chondrocytes, can cause a variety of spinal diseases, such as spinal stenosis, radiculopathy, and cauda equina syndrome. The ligamentum flavum connects the arch plates of adjacent vertebrae. The ligamentum flavum attaches upward to the front of the adjacent vertebral plate above and downward to the back of the adjacent vertebral plate below; the ligamentum flavum can extend to the intervertebral joint capsule at the lateral attachment site and to the spinous process of the vertebral plate at the medial side. Most of the ligamentum flavum is elastic fibrous tissue, and the fibers of the ligamentum flavum are arranged almost vertically. The front of the ligamentum flavum is covered by a membrane, which has a smooth texture. The ligamentum flavum is thin in the neck, thicker in the thorax, and thickest in the lumbar region. When the spine is flexed forward, the ligamentum flavum limits the separation of the arch plate, aids the forward-flexed spine in maintaining an upright posture, and sometimes protects the intervertebral discs from damage. The medial portion of the ligamentum flavum has small holes at the midline where veins travel.

RETRACTED

As we age, the ligamentum flavum will gradually thicken and proliferate and become less elastic, while degenerative symptoms such as calcification and ossification may occur. Degenerative changes of the ligamentum flavum may cause stenosis of the corresponding spinal canal and may also cause clinical symptoms of nerve root compression in the corresponding segment and spinal cord. The main pathological changes of degenerative ligamentum flavum are ligamentum flavum hypertrophy, ligamentum flavum calcification, and ligamentum flavum ossification. Hypertrophy of the ligamentum flavum refers to the thickening and hyperplasia of the intervertebral ligament, which is caused by a long period of degenerative disease, and due to the location of the ligamentum flavum, hypertrophy of the ligamentum flavum also becomes one of the main causes of intervertebral stenosis. The lesions are more common in the L4 and L5 vertebrae and less common in the thoracic and cervical spine. The cause of ligamentum flavum hypertrophy is thought to be due to gradual fibrosis of the ligament during the process of mechanical stress, inflammatory response, and scar repair, based on aging or mechanical instability of the lumbar spine and poor spinal stability. Thickening of the ligamentum flavum can lead to a narrowing of the corresponding intervertebral canal lumen and a smaller intervertebral foramen, which can produce symptoms of spinal nerve root compression. In some people, as they age or for other reasons, the ligamentum flavum may become excessively thickened, compressing the spinal nerves and producing the corresponding symptoms, which are more common in the lower lumbar spine. As the ligamentum flavum continues to thicken, collagen fibers continue to increase and may even replace the elastic fibers, eventually leading to the formation of fibrous scarring.

## 4. CT-Influenced Interspinous Foraminoscopy

### 4.1. Materials and Methods

Four hundred and forty patients who required CT examination of lumbar vertebrae and lumbar intervertebral discs due to lumbar discomfort in our hospital from January 1, 2018, to May 30, 2018, were selected, of which 197 patients, 77 males and 120 females, with an age distribution of 20–86 years, were found to have sublaminar spines. The mean age was (58.2 ± 3.8) years. Inclusion criteria are as follows: those who underwent CT examination of the spine and those with complete imaging data. Exclusion criteria are as follows: those who had undergone surgery or trauma to the corresponding lumbar vertebrae, resulting in the destruction of the bony structures of the corresponding vertebrae and lumbar spine attachments. Patients were grouped according to their age: youth group: 20–40 years old; middle-aged group: 41–60 years old; elderly group: 61 years old and above. The grouping was done according to the different segments of the vertebral body. The vertebrae were grouped according to their degree of stability and divided into the stable spine (control group) and unstable spine (observation group). The unstable spine group included the following: those with scoliosis, those with small joint asymmetry, those with a history of trauma to the spine, and those with lumbar spondylolisthesis.

RETRACTED

CT scans of the lumbar spine were performed using Siemens 128-layer spiral CT on all examiners. Patients were placed on the scanning table in a normal supine position, and axial volumetric scans of the spine were performed (scanning range from the T10 vertebrae to the S1 vertebrae). The instrument parameters were set to 1.0 pitch, 512 × 512 matrix, and 0.625 mm layer thickness, and the data were reconstructed in coronal, sagittal, and oblique positions using thin layer scans.

For patients with a sublaminar spine on CT scan, the images from the CT scan of the patient of interest are transferred to a postprocessing workstation (Vit-rea2.0), the 3D images are reconstructed by computer software, and the soft tissue of the vertebral body is removed from the reconstructed images, so that the lateral posterior wall of the spinal canal, the sublaminar spine, and the internal opening of the spinal canal are fully exposed. This allows the physician to observe the morphology of the sublaminar spine and its adjacent relationship with the intervertebral ligament from a holistic perspective in a more intuitive and accurate manner, as shown in Figure 3.

### 4.2. Incidence of Sublaminar Spines in Spinal Segments

It is generally believed that the vertebral bodies in the thoracolumbar and lower lumbar segments of the spine are under more stress, and the analysis revealed a high incidence of sublaminar spines in the corresponding segments. The incidence of different spinal segments was tested by *χ*2 test and the results were statistically significant (*P* < 0.05). See Figure 4 for details.

The concept of spinal stability assumes that under normal physiological conditions the structures of the spine are able to maintain normal structural relationships with each other, maintaining a relatively stable relationship that does not produce compression and damage to the spinal cord or spinal nerve roots, thereby causing clinical symptoms. Factors affecting spinal stability generally include four major categories: structural stabilizers (shape and size of the vertebral body), shape, size, and orientation of the articular surfaces; dynamic stabilizers which are ligaments, fibrous rings, and articular surface cartilage; hydrodynamic stabilizers which are the expansion of the nucleus pulposus; and random stabilizers which are overall motor and local stabilizing muscles.

RETRACTED

Pathological changes in the above four factors can cause a decrease in spinal stability, such as spinal fractures leading to the destruction of structural stabilizers and lumbar sprains resulting in damage to the dynamic stabilizers; accompanied by age, the expansion of the nucleus pulposus will gradually decline, as well as there will be a decline in muscle function. Therefore, the author identifies scoliosis, small joint asymmetry, a history of trauma to the spine, and lumbar spondylolisthesis as the unstable spine. The incidence of the sublaminar spine in the unstable spine group was higher than the incidence of the sublaminar spine in the stable spine group, and the *P* < 0.05 for both groups was statistically significant, as shown in Figure 5.

## 5. Results and Discussion

The sublaminar spine is a spine-like bony protrusion that occurs at the junction of the anterior and inferior lateral margins of the vertebral plate with the root of the inferior articular eminence and above and is located on the anterolateral side of the outer edge of the intervertebral ligament, with varying morphology and irregular margins, mostly wide at the top and narrow at the bottom, and with a still smooth surface. From the morphological-anatomical point of view, the sublaminar spine can be considered as a bony protrusion located on the vertebrae of the spine, and most of the structures are irregular and have different morphologies, including spine, unimodal, and multifidus types. The sublaminar spine is relatively stable, located on the anterolateral side of the outer edge of the ligamentum flavum of the spinal canal, at the junction between the root of the subacromial synapse and the anterolateral edge of the vertebral plate, with a downward-pointing bony prominence. The distribution of the inferior spine of the vertebral plate varies from patient to patient and may show a single vertebral unilateral, single vertebral bilateral, jumping, segmental, or continuous distribution. Because its lower narrower tip points to the intervertebral canal or spinal canal, it participates in the bony posterior wall that constitutes the spinal canal and intervertebral canal, often causing compression of nerves within the patient's spine or triggering the spinal canal compression phenomenon known as a dural sac in the spine. The sublaminar spine is clearly visible on CT, but it is barely visible on conventional radiographs, mainly due to its location and structure. The sublaminar spine is located above the root of the inferior synovial process and at the junction of the anterior and inferior lateral margins of the vertebral plate, which is difficult to visualize on conventional radiographs due to the overlap of bony structures. By using the image information to reconstruct the relevant coronal, sagittal, and oblique positions as well as to reconstruct the 3D image, the influence of the overlapping bony structures on the observed diagnostic results can be almost completely eliminated, and the position, morphology, and adjacent relationship with the surrounding structures of the sublaminar spine can be displayed more visually and accurately, as shown in Figure 6, giving the physician a more intuitive, holistic, and comprehensive understanding of the structure. The incidence of the sublaminar spine was studied by dividing the patients into three groups according to age groups: young, middle-aged, and old. After data analysis, it was found that the incidence of the sublaminar spine was significantly higher in the middle-aged and elderly groups than in the young group. This indicates that the incidence of the sublaminar spine increases with age, and it is inferred that the occurrence of the sublaminar spine may be related to age and degenerative changes of the spine.

RETRACTED

The higher incidence and larger morphology of sublaminar spines in the lower thoracic segment may be due to the greater mobility and weight bearing of the small joints at the lower thoracic segment, and this distribution is similar to the distribution pattern of ossification of the ligamentum flavum in the thoracic and lumbar spine as reported. In the author's study, further observation and comparison of different vertebral bodies in patients with sublaminar spines revealed that sublaminar spines mainly occurred in the T11-L5 segment of the patient's spine, with the highest incidence of sublaminar spines in T12, followed by T11, L1, L5, L2, and L4, respectively, with decreasing incidence of sublaminar spines in L3 in that order. In this study, the incidence of the sublaminar spine was the highest in the T12, T11, L1, and L5 vertebrae of the thoracolumbar and lower lumbar segments, so it can be considered that the occurrence of the sublaminar spine is related to the stress effect, as shown in Figure 7. According to the stability of the vertebral body, the spine was divided into the unstable spine group and the stable spine group during the analysis, and the results of the study showed that the incidence of sublaminar spines in the unstable spine was significantly higher than the incidence of sublaminar spines in the stable spine and was statistically significant, indicating that the formation of sublaminar spines is likely to be related to the uneven stress on the spine. Therefore, it is considered that the formation of sublaminar spines may be related to the degeneration and stress of the intervertebral ligament. There is no uniform understanding of the mechanism of sublaminar spine formation, and there are two different views. One view is that the sublaminar spine is a bony protrusion formed by the ossification of the lateral part of the intervertebral ligament.

RETRACTED

The main basis of the above view is that the marginal part of the sublaminar spine is consistent with the lateral edge of the intervertebral ligament, and the ossification of the intervertebral ligament occurs mainly in the small joints with high mobility, such as the vertebral body in the thoracolumbar segment, and the sublaminar spine also occurs there, which is consistent with the distribution pattern of the incidence of the sublaminar spine. The pathogenesis is not yet clear, but studies have shown that calcification and ossification of the ligamentum flavum are positively correlated with age, small joint degeneration, and stress. The sublaminar spine is closely related to the position of the ligamentum flavum, and its incidence is higher in areas of greater mobility, age, and spinal instability, so it is reasonable to believe that the formation of the sublaminar spine is the result of further proliferation and ossification of the ligamentum flavum based on degeneration, strain, repeated repair, and hyperplasia. Another view is that the sublaminar spine is a bony structure that normally occurs in the adult spine and is the attachment point of the intervertebral ligamentum flavum to the vertebral plate. This view is based on the fact that the sublaminar spine is more fixed and connected to the intervertebral ligament, so it is considered to be a normal bony structure as an attachment point of the intervertebral ligament on the vertebral plate. However, the formation and development of bone tissue do not occur out of thin air but require certain material and physiological mechanisms. The formation of the bone requires the continuous division and proliferation of mesenchymal cells, which will first form an ossification center at the site where bone tissue is expected to form, and the mesenchymal cells in the ossification center will differentiate into osteogenic cells, which will then continue to divide and proliferate and differentiate into osteoblasts, which will form new bone tissue. It can be seen that the growth and occurrence of bone must require the formation of an ossification center, but the author reviewed the relevant data and did not find that the lumbar vertebral body has an obvious ossification center associated with the inferior spine of the vertebral plate during development, which naturally does not become the bony structure of the lumbar vertebral body. Therefore, the author's study supports the first view that the sublaminar spine of the lumbar spine may be a bony protrusion formed during the degenerative disease of the intervertebral ligament and repeated repair and proliferation.

RETRACTED

## 6. Conclusion

In this paper, human behavior recognition algorithm based on optical flow and depth motion map is implemented for action and 3D behavior recognition along the line of sight. The research of this paper is based on three independent recognition flows of Les net 101 (spatial flow, time flow, depth flow) network, and the color information input to the spatial flow network channel is directly processed by a full sampling of the RGB video sequence. And four data expansion methods apply. The optical flow information input to the global flow network channel is extracted from the RGB video sequence using the tv-l1 optical flow algorithm, and the horizontal and vertical components of the tv-l1 optical flow are adjusted. Set 0 to 0 and set all values greater than 255 to 255. DMM computations capture depth motion maps of depth action sequences and effectively capture motion features from projection views on three orthogonal Cartesian planes.

## Figures and Tables

**Figure 1:** Distribution of the sublaminar spine in relation to symptoms.

**Figure 2:** Changes in the exposure rate of dura and nerve roots during interspinous foraminoscopy.

**Figure 3:** CT influences the course of assisted interspinous foraminoscopy.

**Figure 4:** Incidence of the sublaminar spine in patients with a sublaminar spine in different spinal segments.

**Figure 5:** Incidence of sublaminar spines in stable and unstable spines.

**Figure 6:** Relationship between the sublaminar spine and the ligamentum flavum.

**Figure 7:** Comparison of the incidence of sublaminar spines at the vertebral body.

## Data Availability

The data used to support the findings of this study are available from the corresponding author upon request.
